RETRACTED

# Utilization of Artificial Neural Network in Predicting the Total Organic Carbon in Devonian Shale Using the Conventional Well Logs and the Spectral Gamma Ray

**DOI:** 10.1155/2021/2486046

**Published:** 2021-07-22

**Authors:** Osama Siddig, Ahmed Abdulhamid Mahmoud, Salaheldin Elkatatny, Pantelis Soupios

**Affiliations:** ^1^Department of Petroleum Engineering, King Fahd University of Petroleum & Minerals, Dhahran 31261, Saudi Arabia Box 5049; ^2^Department of Geosciences, King Fahd University of Petroleum & Minerals, Dhahran 31261, Saudi Arabia Box 5049

## Abstract

Due to high oil and gas production and consumption, unconventional reservoirs attracted significant interest. Total organic carbon (TOC) is a significant measure of the quality of unconventional resources. Conventionally, TOC is measured experimentally; however, continuous information about TOC is hard to obtain due to the samples' limitations, while the developed empirical correlations for TOC were found to have modest accuracy when applied in different datasets. In this paper, data from Devonian Duvernay shale were used to develop an optimized empirical correlation to predict TOC based on an artificial neural network (ANN). Three wells' datasets were used to build and validate the model containing over 1250 data points, and each data point includes values for TOC, density, porosity, resistivity, gamma ray and sonic transient time, and spectral gamma ray. The three datasets were used separately for training, testing, and validation. The results of the developed correlation were compared with three available models. A sensitivity and optimization test was performed to reach the best model in terms of average absolute percentage error (AAPE) and correlation coefficient (*R*) between the actual and predicted TOC. The new correlation yielded an excellent match with the actual TOC values with *R* values above 0.93 and AAPE values lower than 14%. In the validation dataset, the correlation outperformed the other empirical correlations and resulted in less than 10% AAPE, in comparison with over 20% AAPE in other models. These results imply the applicability of this correlation; therefore, all the correlation's parameters are reported to allow its use on different datasets.

## 1. Introduction

As oil and gas production and consumption continue, this leads to the gradual diminishing of conventional hydrocarbon reserves worldwide. Hence, the daily oil production rate from currently producing reservoirs considerably declined [1, 2]. Therefore, recently source rock and unconventional reservoirs attracted significant interest [3, 4]. Exploration of unconventional resources is more complicated than the exploration of conventional reservoirs because they are more complex, tight, and impermeable [5].

RETRACTED

Recently, the source rock reservoirs such as shale reservoirs were extensively discovered in many countries, including the United States, Canada, China, Argentina, Saudi Arabia, United Arab Emirates, and Algeria; as a consequence, this resulted in a significant increase in the discovered hydrocarbon resources [6, 7].

Compared to the conventional reservoirs, the unconventional resources are self-generating and self-storing reservoirs; so, it is notoriously critical that the hydrocarbon generation potential of these kinds of reservoirs be evaluated. In addition, the unconventional resources are also costly to develop, not easy to extract the hydrocarbon from these resources, and notoriously difficult to define the reservoir (i.e., net pay). This confirms the importance of evaluating the ability of the unconventional resources for hydrocarbon generation in a cost-effective manner with high accuracy [4, 6].

One of the most powerful and effective reservoir parameters that indicate the potential of hydrocarbon generation and evaluate the quality of the unconventional resources is the total organic carbon (TOC) [8], which several experts and studies had previously considered to assess the potential of hydrocarbon generation [9–11].

In general, TOC content is measured in the laboratory by conducting the rock pyrolysis experiment [12, 13]. Due to the high cost of the experiments, there is a limitation on the number of samples evaluated at the laboratory. It is a costly and challenging process to have an experimentally continuous TOC estimation in the targeted formations, which affects the subsequent evaluation of the unconventional resources [14].

However, several previous empirical correlations and artificial intelligence models for TOC determination were developed based on the continuous well logs and measured TOC determined from laboratory experiments using a limited number of core samples or drilled cuttings. Then, the developed correlation could be used to reliably calculate the TOC for multiple wells [15–19].

### 1.1. Empirical Correlations for TOC Estimation

Schmoker [20] developed the first empirical equation for TOC prediction, that is, in equation (1), this model was developed for Devonian shale and it predicts the volume percentage of the TOC based on the organic matter free rock density (*ρ*_*B*_) and the bulk formation density (*ρ*); then, the weight percentage of the TOC could be calculated as explained by Schmoker [20]:

(1) $$\begin{array}{c} \text{TOC}\left(\text{vol}.\%\right)=\frac{\left(\rho_{B}-\rho \right)}{1.378}, \end{array}$$

where *ρ*_*B*_ and *ρ* are both in g/cm^3^.

RETRACTED

Schmoker [21] presented a revised form equation (1) to be applied in Bakken shale; this revised form is presented in equation (2), and it calculates the TOC content as the weight percentage based on the organic matter density (*ρ*_*o*_), the organic matter-to-organic carbon ratio (*R*), and grain and pore fluid average density (*ρ*_mi_):

(2) $$\begin{array}{c} \text{TOC}\left(\text{wt}.\%\right)=\frac{\left[\left(100\rho_{o}\right)-\left(\rho -0.9922\rho_{\text{mi}}-0.039\right)\right]}{\left[\left(R\rho \right)\left(\rho_{o}-1.135\rho_{\text{mi}}-0.675\right)\right]}, \end{array}$$

where *ρ*_*o*_ and *ρ*_mi_ are in g/cm^3^.

In 1990, Passey et al. [22] developed the Δlog*R* model that is nowadays commonly used to evaluate the TOC as a function of the formation resistivity (FR) and sonic transit time logs (Δ*t*). Equations (3) and (4) summarize the Δlog*R* model, which predicts the TOC from the logs separation (Δlog*R*), FR, Δ*t*, the base formation resistivity (FR_baseline_), the base formation sonic transit time (Δ*t*_baseline_), and the level of maturity (LOM):

(3) $$\begin{array}{c} \Delta \;\log\;R\;=\;\log_{10}\left(\frac{\text{FR}}{{\text{FR}}_{\text{baseline}}}\right)+0.02\times \left(\Delta t-\Delta t_{\text{baseline}}\right), \end{array}$$

(4) $$\begin{array}{c} \text{TOC }=\;\Delta \;\log\;R\;\times 10^{\left(2.297-0.1688\times \text{LOM}\right)}, \end{array}$$

where FR and FR_baseline_ are in ohm.m and Δ*t* and Δ*t*_baseline_ are in *μ*s/ft.

Charsky and Herron [23] evaluated the accuracy of Schmoker and ∆log*R* models in estimating the TOC for different formations in four various wells. Charsky and Herron [23, 24] reported that both models are not highly accurate, and they predicted the TOC with a high average absolute difference from the actual TOC.

Several recent studies focused on enhancing the predictability of the Δlog*R* model in estimating the TOC [11, 24, 25]. Wang et al. [26] developed a revised ΔlogR model to estimate the TOC for Devonian shale from the FR, Δ*t*, RHOB, and gamma ray (GR). In Wang's model, Δlog*R* is calculated by equation (5) or (6), while the TOC is calculated by equation (7). The authors reported that the accuracy of the Δlog*R* model was improved after including the gamma ray. They also simplified using the ΔlogR model by replacing the LOM on the original model with the vitrinite reflectance (*R*_*o*_) or *T*_max_, which also decreased the practical problems [27]:

(5) $$\begin{array}{c} \Delta \;\log\;R\;=\;\log_{10}\left(\frac{\text{FR}}{{\text{FR}}_{\text{baseline}}}\right)+\frac{1}{\ln\;10}\frac{m}{\Delta t-\Delta t_{m}}\times \left(\Delta t-\Delta t_{\text{baseline}}\right), \end{array}$$

(6) $$\begin{array}{c} \Delta \;\log\;R\;=\;\log_{10}\left(\frac{\text{FR}}{{\text{FR}}_{\text{baseline}}}\right)+\frac{1}{\ln\;10}\frac{m}{\rho_{m}-\rho }\times \left(\rho -\rho_{\text{baseline}}\right), \end{array}$$

(7) $$\begin{array}{c} \text{TOC }=\left[\alpha \Delta \;\log\;R+\beta \left(\text{GR}-{\text{GR}}_{\text{baseline}}\right)\right]\times 10^{\left(\delta +\eta \;T_{\max}\right)}, \end{array}$$

where *T*_max_ is the indicator of maturity in °C, *m* is the exponent of cementation, Δ*t*_*m*_ is the matrix sonic transit time, *α*, *β*, *δ*, and *η* are constants, other parameters are with the same definitions as in equations (1) to (4), and units are consistent between all the equations.

RETRACTED

In another study, Wang et al.'s [26] models were revised by Zhao et al. [28] to develop empirical correlations for TOC estimation. These models do not depend on the LOM, vitrinite reflectance (*R*_*o*_), or *T*_max_. These models account for the TOC based on the FR, bulk gamma ray (GR), and Δ*t* or bulk formation density (RHOB) logs.

### 1.2. Evaluation of the TOC Using Artificial Intelligence

The empirical correlations discussed in the previous section yield low-accuracy predictions when used with different datasets. Recently, several authors evaluated the use of the powerful nonlinear fitting abilities of the artificial intelligence (AI) techniques in predicting the TOC [29, 30].

Kadkhodaie-Ilkhchi et al. [31] developed a committee machine with an intelligent system (CMIS) to evaluate the TOC from the well-log data of the GR, FR, Δ*t*, RHOB, and neutron porosity (CNP). The CMIS was constructed using the genetic algorithm having as inputs the TOC values estimated with the neuro-fuzzy (NF), fuzzy logic (FL), and backpropagation neural network (NN).

Another TOC model was developed by Zhu et al. [30] using the support vector machine (SVM) to evaluate the TOC from the well-log data. This model predicted the TOC with high accuracy compared with the Δlog*R* model.

Shi et al. [32] compared the predictability of the extreme learning machines (ELM) and artificial neural network (ANN) model in predicting the TOC based on the combination of GR, RHOB, CNP, compressional wave slowness (DTC), and spectrum logs of uranium (Ur), thorium (Th), and potassium (K). This study showed that the ELM model is most accurate in predicting the TOC when compared with the ANN.

Mahmoud et al. [9, 33] were the first to extract an empirical correlation out of the optimized ANN model to evaluate the TOC from the well logs of the FR, GR, RHOB, and Δ*t*. This extracted correlation converts the ANN model to a white box which could then be easily applied to the new data. The developed correlation also overperformed all the available correlations for TOC prediction. Later on, Elkatatny [34] optimized the ANN model using the self-adaptive differential evolution algorithm, and he developed another model for TOC prediction based on the optimized ANN model. Elkatatny [34] proved that his correlation improved the predictability of the Mahmoud et al. [9, 33] correlation.

RETRACTED

Mahmoud et al. [17] developed two TOC prediction models based on the SVM and functional neural networks. The authors reported that the FNN model overperformed the SVM in TOC prediction, and no correlation was extracted from these optimized models.  Table 1 summarizes different research studies that employed artificial intelligence techniques to predict the TOC from well logs.

In this study, a new optimized ANN-based empirical correlation is developed to predict the TOC of shales from the well logging data such as formation resistivity, sonic transient time, bulk density, bulk gamma ray, neutron log porosity, and spectral gamma-ray logs of Ur, Th, and K. The parameters of the model are presented to allow the interested researcher or companies to utilize.

## 2. Methodology

In this study, a correlation was developed based on the extracted parameters of the optimized artificial neural network (ANN) model to estimate the TOC as a function of eight well logs of the FR, Δ*t*, RHOB, CNP, GR, and spectral gamma-ray logs of the Ur, Th, and K. The following sections explain the different steps for optimizing the ANN model, extraction of the empirical correlation, and validation of the developed correlation.  Figure 1 summarizes the methodology applied in this research work.

### 2.1. Data Description

The eight input well logs and their corresponding TOC were collected from three different wells in Devonian Duvernay shale, and 891 datasets from Well-A were used to learn the ANN model. In contrast, 291 datasets from Well-B and 82 datasets from Well-C were used to test and validate the developed empirical equation.

Devonian Duvernay shale is a well-known organic-rich source rock in the Western Canada Sedimentary Basin [44]. This shale formation is liquid-rich and contains 61.7 billion barrels of oil in place and 443 Trillion cubic feet of gas in place [45].

### 2.2. Core Samples Collection and Testing

The actual TOC values considered to train the ML algorithms were obtained based on lab measurements conducted on drilling cuttings. The collected cuttings were analyzed using Rock-Eval 6. Before testing, the samples were grinded to a small size (<63 *μ*m). Then, the samples were thermally decomposed using a pyrolysis oven to evaluate the pyrolyzable carbon and mineral carbon for all samples as a weight percentage of the total sample. Then, the samples were burned at 300°C for 30 seconds in the oxidation oven to determine the residual carbon and oxidized mineral-carbon weight percentages. More discussions and details of the considerations and sample preparation for testing through Rock-Eval 6 were provided by different authors [46].

RETRACTED

### 2.3. Well Logs

In well logging, the in situ properties of rocks around the wellbore are indirectly estimated from electric, acoustic, and nuclear indicators. The interpretations of these indicators reflect the existence of hydrocarbon, petrophysical properties, and lithology of the formation [47, 48]. In this study, the following well logs' records were used:

  Formation resistivity (FR): it is a measure of electrical resistivity in three increasing depths from the well which is mainly interpreted to know the fluids' saturations, and hence, the existence of hydrocarbon [49, 50].
  Sonic log: it is a measure for the time required for a sound wave to travel for a predetermined distance, which depends on the matrix elasticity and porosity [51]; therefore, it is used in the identification of lithology, fractures, and porosity.
  Density log: it is a record of the bulk density around the well; this density measure covers the matrix and the pores filled with fluid, which can be used to quantify the porosity fraction.
  Neutron log: it is a log relying on a neutron source to measure the hydrogen index, and consequently, the porosity of the formation.
  Gamma-ray log: it measures the natural gamma radiations, and thus, it is used to distinguish shales from other sedimentary rocks.
  Spectral gamma-ray log: it is a sophisticated measure for gamma ray that uses the energy of gamma rays and identifies the elements that emitted them.

### 2.4. Data Preprocessing

Before training the ANN model, the datasets were preprocessed to remove any nonviable data and outliers. All zeroes or unrealistic values were removed from the input datasets. The outliers (their values differ significantly from the other data points, by at least three times the standard deviation, SD) were also removed from the training dataset. The statistical characteristics of the training data (i.e., the 891 data points of Well-A) are summarized in Table 2.

### 2.5. Optimization of the Artificial Neural Network Model

ANN is a popular machine-learning method that mimics the brain's neurons that could be utilized in clustering, classification, or regression [52, 53]. ANN contains various parameters such as neurons, activation functions, layers, and learning functions. Many successful implementations of ANN in the oil sector have been reported [54–58].

RETRACTED

The ANN model was trained and optimized in this work using the 891 data points of the eight different input parameters collected from Well-A to estimate the TOC. These input parameters include FR, Δ*t*, RHOB, CNP, GR, and spectral gamma-ray logs of the Ur, Th, and K.  Figure 2 shows the well logs collected for the training of the ANN model.

The performance of different parameters inside the ANN algorithm was evaluated by conducting sensitivity analysis during the optimization stage. These studied parameters include the number of neurons in each layer, number of layers, type of the network function, and training and transfer functions. The algorithm's design parameters were tested by running the algorithm inside *for*-loops in the MATLAB software to evaluate several parameters' combinations.

### 2.6. Testing and Validation of the Developed Model

The accuracy of the developed model was tested on 291 data points and validated on 82 data points collected from Well-B and Well-C, respectively. The location of these two wells is relatively close to the training well. The performance ANN predictions were also compared with currently available correlations, namely, Schmoker model, Δlog*R* method, and Zhao et al. [28] correlation.

## 3. Results and Discussion

### 3.1. Training the Artificial Neural Networks

The ANN model was trained for TOC estimation based on eight well-log data of FR, Δ*t*, RHOB, CNP, GR, and spectral gamma-ray logs of the Ur, Th, and K. The training dataset consisted of 891 data points from Well-A.  Figure 3 compares the actual and predicted TOC for the training dataset. It should be noticed in Figure 3(a) that the profiles of actual and estimated TOC match each other entirely with a correlation coefficient of 0.98 and an average error of 8.8%.  Figure 3(b) shows the cross plot of the given and the predicted values, which confirm the model's accuracy since all the points are near the 45° line.

### 3.2. Model Testing

The accuracy of the initial model was confirmed using the TOC estimations from the additional unseen 291 data points from Well-B.  Figure 4 shows the actual and ANN-predicted TOC for the testing dataset. The ANN-based model resulted in 0.93 and 14% correlation coefficient, respectively, for the testing dataset. Similar to the training results, the profile of the estimated values follows the same trend as the actual values, as seen in Figure 4(a). Likewise, in Figure 4(b), most of the points in the cross plot fall close to the 45° line.

### 3.3. ANN-Based Empirical Correlation

A sensitivity analysis has been applied, and an optimized model based on two evaluation criteria, the correlation coefficient (*R*) and the average absolute percentage error (AAPE), was developed. The different sets of inputs that have been tested to find the best TOC predictions are presented in Table 3.

RETRACTED

Table 3 shows that the highest prediction accuracy was achieved when all eight logs were used, while the lowest performance happened when GR and spectral GR were excluded. The optimum ANN parameters for the inputs' set that yielded the best fitting are reported in Table 4.

As shown in Table 3, the best fit was obtained using the tan-sigmoid transfer function, which results in correlation coefficients of 0.98 and 0.93 in training and testing, respectively, with AAPE values not more than 14%. The generated model is expressed by equation (8), while Table 5 shows the weight and biases that are used in the model:

(8) $$\begin{array}{c} \text{TOC}=\left[\sum_{i=1}^{N}W_{2,i}\left(\frac{1}{1+e^{-\left(W_{11,i}*\text{FR}+W_{12,i}*\Delta T+W_{13,i}*\text{RHOB}+W_{14,i}*\text{CNL}+W_{15,i}*\text{GR}+W_{16,i}*\text{Ur}+W_{17,i}*\text{Th}+W_{18,i}*\text{Th}+b_{1,i}\right)}}\right)\right]+b_{2}. \end{array}$$

### 3.4. Model Validation and Results Comparison

The previous results indicate a good accuracy of the model developed in this study in estimating the TOC in Devonian shale. The dataset of 82 data points from another well (Well-C) has been used to validate the new correlation. Well-C is located in the vicinity of the Well-A and Well-B that have been used for training and testing, the validation dataset covers a depth interval of over 140 ft. The prediction accuracy of equation (8) was compared with three of the available models for TOC prediction, namely, Schmoker model, Δlog*R* method, and Zhao et al. [28] correlation.

Figure 5 compares the accuracy of the TOC prediction for all these models and correlations for the validation data of Well-C. As shown in Figure 5, the new correlation outperformed all other correlations in estimating the TOC with AAPE of only 9.7% and high *R* of 0.97, while Zhao et al. [28] correlation was the second accurate, and it estimated the TOC with AAPE and *R* of 20.2% and 0.84, respectively. The Δlog*R* method calculated the TOC with high AAPE of 24.6% and low *R* of 0.83, and the least accurate model was the one developed by Schmoker which predicted the TOC with the highest AAPE of 48.6% and the lowest *R* of 0.80. Visual comparison of all plots of Figure 5 also confirmed the high accuracy of equation (8) compared to the other models.

The previous results and analysis confirm the accuracy of the developed equation in predicting the TOC for Devonian shale. This equation estimated the TOC from the conventional well logs and spectral gamma-ray logs. It overperformed the current empirical equations, which calculated the TOC based on RHOB log only (Schomoker model), or a combination of FR and Δ*t* logs and LOM (Δlog*R* method), or bulk gamma ray, FR, and Δ*t*, or RHOB logs (Zhao et al. [28] correlation). Comparing different (previous) applied models for TOC estimation, the suggested one from this work proves the applicability of the developed correlation for TOC prediction in Devonian shale.

RETRACTED

### 3.5. Model's Limitations

The data used in this research work have been gathered from three wells in the same field. The data were also limited to Devonian shale. Therefore, the accuracy of this model is not guaranteed if used in a different type of formation or different data ranges other than the one presented in this study.

## 4. Conclusions

In this study, an optimized ANN-based empirical correlation for TOC prediction in Devonian Duvernay shale from conventional well logs and spectral gamma-ray logs was developed based on the optimized ANN model. The findings reported in this paper are summarized as follows:

- The ANN model predicted the TOC for the training and testing datasets with AAPE and *R* of 8.8% and 0.98 for training and 14% and 0.93 for testing.
- The validation dataset of 82 data points from the third well was completely hidden from the ANN algorithms. This model yielded a 0.97 correlation coefficient and 9.7% AAPE in this dataset.
- The validation dataset was also used to compare the performance of the developed empirical correlation with three different empirical correlations for TOC prediction. The model significantly outperformed the other models with correlation coefficients less than 0.85 and AAPE over 20%.
- The weights and biases of the developed model are all presented in this paper, which will facilitate its use with similar datasets.

## Figures and Tables

**Figure 1:** Methodology flowchart.

**Figure 2:** The well logs of FR, Δ*t*, RHOB, CNP, GR, and spectral gamma-ray logs of the Ur, Th, and K used to train the ANN model.

**Figure 3:** The actual and predicted TOC for the training dataset. (a) Profiles with Well-A depth index. (b) Cross plot around 45° line.

**Figure 4:** The actual and predicted TOC for the testing dataset. (a) Profiles with Well-B depth index. (b) Cross plot around 45° line.

**Figure 5:** Comparison of the prediction accuracy of Schmoker model, Δlog*R* method, Zhao et al. [28] correlation, and equation (8), using the validation dataset of Well-C.

**Table 1:** Summary of different research studies that employed AI techniques to predict the TOC.

Ref.	AI method (s)	Accuracy (*R*^2^)	Data points	Inputs	Formation/basin
[9]	ANN	0.89–0.93	442	FR, Δ*t*, RHOB, and GR	Barnett and Devonian shale formations
[10]	CNN	0.8303	125	FR, Δ*t*, RHOB, CNP, and GR	Shahejie Formation
[31]	FL, NF, and NN	0.845	124	FR, Δ*t*, RHOB, CNP, and GR	Kangan-Dalan Formation
[35]	ANN	0.89	78	FR, Δ*t*, GR, Th, and K	Kazhdomi and Kangan-Dalan Formations
[36]	GPR	NA	NA	FR, Δ*t*, RHOB, CNP, GR, Ur, Th, and K	Ordos basin and Canning basin
[37]	ANN and FL	0.776–0.992	2875	FR, Δ*t*, RHOB, and CNP	Gadvan Formation
[38]	ANN	NA	200	FR, Δ*t*, CNP, GR, Th, and K	Kazhdomi and Kangan-Dalan Formations
[14]	FL	0.9425	31	FR, Δ*t*, RHOB, CNP, GR, Ur, Th, and K	Kazhdumi Formation
[39]	ANN	0.98	70	FR and Δ*t*	
[40]	ANN	0.963	54	FR, Δ*t*, RHOB, CNP, and GR	Khatatba and Ras Qattara Formations
[41]	SVM	0.75	18	FR, Δ*t*, RHOB, SP, and GR	Beibu Gulf basin
[29]	SVM	0.69	31	FR, Δ*t*, RHOB, CNP, GR, Ur, Th, and K	Jiumenchong Formation
[32]	ELM and ANN	0.87–0.91	185	FR, Δ*t*, RHOB, CNP, GR, Ur, Th, and K	Sichuan Basin
[42]	ANN and SVM	0.9–0.927	215	FR, SP, Δ*t*, RHOB, CNP, GR, Ur, Th, and K	Tonghua Basin
[34]	ANN	0.98	460	FR, Δ*t*, RHOB, and GR	Barnett and Duvernay shales
[17]	FNN and SVM	0.74–0.77	+500	FR, Δ*t*, RHOB, and GR	Devonian and Barnett shales
[33]	ANN	0.93	442	FR, Δ*t*, RHOB, and GR	Barnett shale
[18]	FL	0.91	645	FR, Δ*t*, RHOB, and GR	Barnett shale
[43]	ANFIS, FNN, and SVM	0.82–0.870	+800	FR, Δ*t*, RHOB, and GR	Barnett shale

RETRACTED

**Table 2:** The statistical description Well-A dataset.

Statistical parameter	FR (Ω.m)	Δ*t* (*μ*sec/ft)	RHOB (g/cm^3^)	CNP	GR (API)	Ur (wt. %)	Th (ppm)	K (ppm)	TOC (wt. %)
Minimum	3.71	51.0	2.39	0.019	22.9	1.39	1.97	0.130	0.76
Maximum	1675	96.6	2.77	0.346	298	22.6	17.0	4.06	5.66
Mean	110	77.9	2.545	0.174	95.5	6.16	9.01	1.51	2.78
Median	43.0	79.0	2.535	0.174	100	5.7362	9.1181	1.47	2.74
Standard deviation	176	8.56	0.075	0.052	38.9	3.16	2.517	0.607	1.30
Sample variance	30890	73.4	0.006	0.003	1510	9.96	6.337	0.368	1.69
Kurtosis	21.8	0.227	−0.465	0.984	3.43	6.81	0.315	1.14	−1.08
Skewness	3.98	−0.630	0.436	−0.127	0.837	2.13	-0.135	0.554	0.181

**Table 3:** The optimum ANN parameters.

Inputs' set	AAPE (%)	*R*
FR, Δ*t*, RHOB, and CNP	24.6	0.83
FR, Δ*t*, RHOB, CNP, and GR	15.2	0.92
Δ*t*, RHOB, CNP, GR, Ur, Th, and K	11.0	0.96
FR, RHOB, CNP, GR, Ur, Th, and K	8.92	0.97
FR, Δ*t*, CNP, GR, Ur, Th, and K	11.6	0.96
FR, Δ*t*, RHOB, GR, Ur, Th, and K	13.5	0.95
FR, Δ*t*, RHOB, CNP, GR, Ur, Th, and K	8.83	0.98

**Table 4:** The optimum ANN parameters.

Parameter	Value
Number of layers	1
Number of neurons	30
Training function	Bayesian regularization backpropagation (trainbr)
Transferring function	Tan-sigmoid (tansig)

**Table 5:** The weights and biases of the optimized ANN model.

	*W*_11_	*W*_12_	*W*_13_	*W*_14_	*W*_15_	*W*_16_	*W*_17_	*W*_18_	*b*_1_	*W*_2_	*b*_2_
1	0.61	−0.09	0.18	−0.09	0.45	0.26	0.08	0.31	−0.62	0.08	0.87
2	−1.01	0.84	2.94	1.62	1.02	1.83	−2.05	3.09	3.48	4.29	
3	−9.55	−0.03	-4.46	−0.60	−0.56	0.39	0.19	−0.10	−7.91	9.29	
4	0.61	−0.09	0.18	−0.09	0.45	0.26	0.08	0.31	−0.62	0.08	
5	10.93	−5.32	7.04	9.27	1.22	−9.88	0.31	−9.72	4.43	4.79	
6	9.88	3.54	-2.63	−4.99	−3.21	−2.64	6.28	17.86	7.57	−0.04	
7	11.36	−0.76	−3.47	−1.01	1.04	−6.58	4.62	3.01	11.66	−0.65	
8	0.61	−0.09	0.18	−0.09	0.45	0.26	0.08	0.31	−0.62	0.08	
9	3.66	3.26	−5.05	−3.42	0.24	−0.98	−2.75	−0.38	2.44	−5.47	
10	−5.23	−0.29	-0.05	0.46	4.82	5.44	2.82	1.94	2.81	−0.88	
11	5.59	22.15	15.60	8.00	−1.24	7.31	11.57	1.19	−2.36	−0.10	
12	4.14	−4.00	−4.99	−6.21	−2.48	2.39	−3.84	−1.51	7.06	0.12	
13	−10.26	−1.50	-0.35	0.95	3.37	-0.66	−1.85	3.38	−3.72	−11.03	
14	−4.72	−4.24	1.32	−1.48	0.32	7.51	−6.50	−4.41	−2.21	5.70	
15	0.61	−0.09	0.18	−0.09	0.45	0.26	0.08	0.31	−0.62	0.08	
16	0.61	−0.09	0.18	−0.09	0.45	0.26	0.08	0.31	−0.62	0.08	
17	1.84	−4.83	6.76	9.50	−4.21	−9.39	−0.63	−8.22	−2.82	−1.77	
18	−2.11	2.97	−3.16	0.69	3.80	−1.16	−5.94	6.64	1.53	−0.17	
19	0.61	−0.09	0.18	−0.09	0.45	0.26	0.08	0.31	−0.62	0.08	
20	0.61	−0.09	0.18	−0.09	0.45	0.26	0.08	0.31	−0.62	0.08	
21	6.30	−10.76	−4.98	−8.24	−5.02	−0.50	−3.48	−6.19	1.72	−1.57	
22	0.61	−0.09	0.18	−0.09	0.45	0.26	0.08	0.31	−0.62	0.08	
23	−2.73	−2.29	−0.37	1.69	3.87	0.87	−2.94	4.04	3.90	6.49	
24	−0.33	−2.61	−5.04	−4.73	−3.56	1.04	0.63	0.51	0.57	−7.93	
25	−1.40	−1.80	−0.21	−2.47	0.71	2.42	−4.40	−3.66	1.57	−10.97	
26	−15.89	−1.60	0.60	2.61	3.41	−5.53	−0.45	1.73	−12.82	7.75	
27	0.61	−0.09	0.18	−0.09	0.45	0.26	0.08	0.31	−0.62	0.08	
28	−11.09	−1.02	−1.02	−4.15	2.20	2.32	−3.74	−3.99	−7.22	4.05	
29	0.61	−0.09	0.18	−0.09	0.45	0.26	0.08	0.31	−0.62	0.08	
30	4.50	9.14	−0.31	3.47	−10.28	3.24	11.40	-8.30	−3.51	−1.81	

RETRACTED

## Data Availability

The data used to support the findings of the study are included within the article and also available from the corresponding author upon request.

## Abbreviations

AAPE: Average absolute percentage error
ANFIS: Adaptive neuro-fuzzy interference system
ANN: Artificial neural network
CNN: Convolutional neural network
CNP: Neutron porosity
ELM: Extreme learning machine
FL: Fuzzy logic
FN: Functional network
FR: Formation resistivity
GPR: Gaussian process regression
GR: Gamma ray
NF: Neuro-fuzzy
NN: Neural network
*R*: Correlation coefficient
RHOB: Bulk density
SP: Spontaneous potential
SVM: Support vector machine
TOC: Total organic carbon
*ρ*: Density
Δt: Sonic transit time.
